The article "Predictive Analysis of Serum NO, PGI2, and Ox-LDL Levels on Disease Progression in Patients with Lacunar Cerebral Infarction" was retracted in 2023. Reasons: suspected computer-generated content; unreliable results or conclusions; concerns about the data; concerns about the results or conclusions.

# Predictive Analysis of Serum NO, PGI2, and Ox-LDL Levels on Disease Progression in Patients with Lacunar Cerebral Infarction

**DOI:** 10.1155/2022/1221810

**Published:** 2022-04-04

**Authors:** Xiaoxiao Tao, Chenfeng Qiu, Xuewen Feng, Linlin Wang

**Affiliations:** Department of Neurology, The First People's Hospital of Wenling, Wenling, Zhejiang, China 317500

## Abstract

**Objective:**

To analyze and predict the progress of patients with lacunar infarction by analyzing the levels of serum NO, PGI2, and Ox-LDL produced by endothelial cells.

**Methods:**

138 patients with lacunar infarction and 34 healthy people were selected. The selected samples were divided into progressive group, nonprogressive group, and control group for biochemical test and endothelial function test. The levels of serum NO, PGI2, and Ox-LDL were obtained. The observation indexes of different groups were compared for statistical analysis and multivariate logistic regression analysis.

**Results:**

The indexes of LI patients in the nonprogression group were different from those in the control group. The content of Ox-LDL in the nonprogression group was higher than that in the control group, while the indexes of serum NO and PGI2 were lower than that in the control group. The level of Ox-LDL in LI patients in the progressive group was much higher than that in healthy people in the control group seven days after admission, while the levels of serum NO and PGI2 were lower, and the difference of serum on was more obvious. The level of Ox-LDL in the progressive group was much higher than that in the nonprogressive group, while the levels of serum NO and PGI2 in the progressive group were lower, and the level of serum NO was significantly different from that in the nonprogressive group. Ox − LDL > 76.48 U/L, NO > 55.24 ummol/L, and PGI2 > 29.78 ng/L were independent risk factors for the progression of lacunar infarction.

**Conclusion:**

Because the patients with lacunar infarction have endothelium-dependent relaxation disorder, the changes of serum NO, PGI2, and Ox-LDL can be used as the evaluation index of the disease progress of patients with lacunar infarction and can be widely used in clinical detection.

## 1. Introduction

According to the relevant research statistics, because of the high incidence rate, high mortality rate, high disability rate, and high recurrence rate of cerebral infarction, cerebral infarction accounts for second of the global death causes, which not only seriously endangering the life safety and quality of life of patients but also causes heavy social burden, financial burden, and life pressure to society and families. Cerebral infarction can be divided into hemorrhagic cerebral infarction and ischemic cerebral infarction according to the pathogenesis. In this study, lacunar infarction (LI) is a kind of ischemic cerebral infarction, with a high incidence rate, accounting for 20-30% of all cerebral infarction. Studies have shown that more than 20% of LI have a progressive deterioration trend after acute onset. Compared with nonprogressive LI, progressive LI has a higher treatment coefficient.

The article "Predictive Analysis of Serum NO, PGI2, and Ox-LDL Levels on Disease Progression in Patients with Lacunar Cerebral Infarction" was retracted in 2023. Reasons: suspected computer-generated content; unreliable results or conclusions; concerns about the data; concerns about the results or conclusions.

Jiao et al. (2019) in the risk factor analysis of progressive large atherosclerotic cerebral infarction (LAA) showed that the independent risk factors of progressive LAA cerebral infarction include increased total leukocyte count, increased admission systolic blood pressure, increased fibrinogen level, intracranial occlusion, and lung infection [1]. Shen et al. (2021) showed in the clinical value study of acute ischemic stroke (AIS) that the combined detection of Lp-PLA2, LDL-C, HDL-C, hs-CRP, Hcy, and FIB levels can synergistically reflect the degree of cerebral infarction of AIS and can be used as an auxiliary index for the evaluation of the progress of AIS [2]. Gao et al. (2021) in the study on the relationship between serum Vaspin expression and inflammatory factors in patients with progressive cerebral infarction (PCI) showed that the serum Vaspin level in patients with PCI is closely related to inflammatory factors, which may be used as an index for disease diagnosis and clinical monitoring, and provide an important reference for the search for diagnostic indicators and treatment of PCI [3]. Chen (2021) in the study of PCI-related risk factors, diabetes history, fever, white blood cell count, Glu, internal carotid artery stenosis, intracranial artery stenosis, CT early cerebral infarction signs, CWI, and severe cerebral microbleeds (>10 lesions) were independent risk factors for PCI [4]. Zhang (2019) in PCI's risk factors study showed that hypertension, diabetes, hyperlipidemia, homocysteine, and atherosclerosis were independent risk factors for PCI [5].

All the above citations are the causes of different cerebral infarction, but the research contents of the cited literature do not study the disease progression of patients with LI based on the levels of serum nitric oxide (no), PGI2, and low density lipoprotein (Ox-LDL). The innovation of this study is to study the effect of serum NO, PGI2, and Ox-LDL levels on the progression of Li by comparing the differences between progressive LI and nonprogressive LI from three aspects: serum NO, PGI2, and Ox-LDL levels.

## 2. Data and Methods

### 2.1. General Clinical Data of Patients

138 patients hospitalized in our hospital from July 2020 to June 2021 were selected, including 67 progressive patients and 71 nonprogressive patients; there were 92 male patients and 46 female patients; the age distribution of patients was 40-75 years old, with an average age of 61.25 ± 3.64 years; there was no significant difference in age, sex, and education level among all patients (*p* < 0.05), which was comparable. See Table 1 below for detailed general information.

The article "Predictive Analysis of Serum NO, PGI2, and Ox-LDL Levels on Disease Progression in Patients with Lacunar Cerebral Infarction" was retracted in 2023. Reasons: suspected computer-generated content; unreliable results or conclusions; concerns about the data; concerns about the results or conclusions.

Case inclusion: (1) patients with first onset; (2) patients and their families were informed of the study and signed relevant consent forms; (3) patients with complete clinical data; (4) patients who meet the approval requirements of the ethics committee.

Case exclusion: (1) patients with serious heart and lung and other important organ diseases; (2) have a history of serious immune system diseases; (3) half a year history of myocardial infarction; (4) patients with incomplete clinical data.

In Table 1, there was no significant difference in the age, gender, education, and pathogenesis of all patients. Make the following Figure 1 according to the data in the above table.

### 2.2. Research Methods and Observation Indicators

All patients received the same treatment scheme after admission, and 34 healthy people who underwent physical examination in our hospital were selected as the control group, including 19 males and 15 females. The average age was 55.34 ± 7.35 years.

In order to facilitate the grouping of patients with progressive or nonprogressive lacunar infarction, it is necessary to score all patients with neurological deficit (NIHSS). The specific evaluation criteria are determined according to the difference between NIHSS score 7 days after admission and NIHSS score on the day of admission. When the score difference is greater than 2 points, it is the progress group, and when the score difference is less than or equal to 2 points, it is the nonprogress group. Fasting venous blood was collected from the first day of admission for biochemical test and endothelial function test. The contents of serum NO, PGI2, and Ox-LDL were extracted and compared with the data of healthy people in the control group. The scoring criteria of NIHSS are shown in Table 2 below.

There are 11 items in Table 2 to score NIHSS for LI patients. The score range is 0-42 points. The higher the score, the more serious the neurological deficit of the patient. Generally, 0-1 points are normal; 1-4: mild; 5-15: moderate; 15-20: moderate to severe; 21-42 points are severe.

### 2.3. Statistical Methods

All inspection data were collected by SPSS 25.0 statistical software for statistical analysis, and the measurement data are analyzed with $\bar{x}\pm s$ indicates that the counting data is expressed in the number of cases and percentage (%), expressed in *χ*^2^ value and *t* value test, when *p* < 0.05, it means that the data difference is statistically significant. Logistic regression analysis was used to analyze the predictors of disease progression in patients with lacunar infarction.

The article "Predictive Analysis of Serum NO, PGI2, and Ox-LDL Levels on Disease Progression in Patients with Lacunar Cerebral Infarction" was retracted in 2023. Reasons: suspected computer-generated content; unreliable results or conclusions; concerns about the data; concerns about the results or conclusions.

## 3. Results

### 3.1. Comparison of Serum NO, PGI2, and Ox-LDL Results between Nonprogressive Group and Control Group

The serum NO, PGI2, and Ox-LDL of 71 LI patients in the nonprogression group, and patients in the progression group selected according to the NIHSS score were compared with the data of 34 healthy people in the control group. The specific test results are shown in Table 3.

In Table 3, from the data comparison between the two groups, it can be found that various indexes of LI patients in the nonprogress group are different from those in the healthy population in the control group. The content of Ox-LDL indexes in the nonprogress group is higher than that in the control group, while the serum no and PGI2 indexes are lower than that in the control group. Make the following Figure 2 according to the data in the above table.

In Figure 2, it can be clearly seen that there are differences in serum NO, PGI2, and Ox-LDL levels between nonprogressive LI patients and healthy people in the control group. Compared with healthy people, nonprogressive LI patients have more Ox-LDL contents, while serum NO and PGI2 contents are less than healthy people.

### 3.2. Comparison of Serum NO, PGI2, and Ox-LDL between Patients in Progression Group and Control Group

The serum NO, PGI2, and Ox-LDL of 67 LI patients screened by NIHSS score for 1-7 days were compared with the data of 34 healthy people in the control group. The specific test results are shown in Table 4.

In Table 4, the data comparison is similar to that of the nonprogression group, but compared with the data in Table 3, the data difference of the progression group is more obvious. At the same time, the Ox-LDL level of LI patients in the progression group seven days after admission is much higher than that of healthy people in the control group, while the levels of serum NO and PGI2 are lower, and the difference of serum on is more obvious. Make the following Figure 3 according to the data in the above table.

In Figure 3, it can be clearly seen that there is a very obvious difference between the observation and detection indexes of patients with progressive LI and the healthy population in the control group (*p* < 0.05), which shows that the patients with progressive LI can be easily distinguished from the healthy population through these indexes.

### 3.3. Comparison of Serum NO, PGI2, and Ox-LDL Results between Progressive Group and Nonprogressive Group

The serum NO, PGI2, and Ox-LDL data of patients in two different observation groups were compared and analyzed. The specific data are shown in Table 5.

The article "Predictive Analysis of Serum NO, PGI2, and Ox-LDL Levels on Disease Progression in Patients with Lacunar Cerebral Infarction" was retracted in 2023. Reasons: suspected computer-generated content; unreliable results or conclusions; concerns about the data; concerns about the results or conclusions.

In Table 5, according to the observation index data of the progress group and the nonprogress group, there are significant differences between the two groups, and the Ox-LDL content level of the progress group is much higher than that of the nonprogress group, while the serum NO and PGI2 content levels of the progress group are lower, and the serum NO level is significantly different from that of the nonprogress group. Make the following Figure 4 according to the data in the above table.

In Figure 4, we can clearly see the difference between the data of the nonprogressive group and the data of the progressive group. Through the figure, we can see that the Ox-LDL level of patients with progressive LI is higher than that of patients with nonprogressive LI, and the contents of serum NO and PGI2 are lower than those of patients with nonprogressive LI, which shows that the disease progress of patients with lacunar infarction can be evaluated by these indicators. The data of progress group, nonprogress group, and control group were combined to make Figure 5.

In Figure 5, it can be seen that compared with the data of the control group, the serum NO, PGI2, and Ox-LDL levels of patients in both the nonprogression group and the progression group are different, and the data gap in the progression group is larger than that in the nonprogression group, which shows that the disease progress of lacunar infarction can be predicted and analyzed by observing the serum NO, PGI2, and Ox-LDL levels.

### 3.4. Multivariate Logistic Regression Analysis Was Performed on the Factors of Disease Progression in Patients with Lacunar Infarction

Import the test data into SPSS software, conduct multiple regression analysis on the predictive factors of serum NO, PGI2, and Ox-LDL, and get the following Table 6.

In Table 6, the variables with statistical comparison differences and their assignment in the univariate analysis of each observation index are explained. According to the multivariate logistic regression analysis, when Ox − LDL > 76.48 U/L, NO > 55.24 ummol/l, and PGI2 > 29.78 ng/l are independent risk factors for the disease progression of patients with lacunar infarction.

## 4. Discussion

According to the previous literature, the incidence rate of lacunar infarction increases with age, and more than 15% of lacunar infarction may cause cerebral palsy or dementia. More than 20% of patients with lacunar infarction may have cerebral infarction again within 5 years of rehabilitation, which indicates the harmfulness of lacunar infarction to human. Therefore, this study predicts and analyzes the disease progress of lacunar cerebral infarction from the bioactive substances produced by endothelial cells, in order to judge the patient's condition through the detection of these bioactive substances.

The article "Predictive Analysis of Serum NO, PGI2, and Ox-LDL Levels on Disease Progression in Patients with Lacunar Cerebral Infarction" was retracted in 2023. Reasons: suspected computer-generated content; unreliable results or conclusions; concerns about the data; concerns about the results or conclusions.

Zhang et al. (2019) showed that TG > 2.2 mmol/l, pro > 45.3 mg/l, and Ox − LDL > 0.75 mg/l were independent risk factors for the disease progression of patients with acute lacunar infarction, which could be used as an observation index to find the disease progression of patients [6]. The conclusion of this study is consistent with this study, but this study only studies the comparison between progressive patients and nonprogressive patients, and this study also sets the data of healthy population as the control group, which increases the credibility of the data. Xu et al. (2020) showed that weight, drinking history, TG, and Hcy are independent risk factors for the development of patients with hypertension complicated with LI. Maintaining normal BMI, limiting alcohol intake, and reducing plasma triglyceride and homocysteine levels may be of positive significance to prevent or reduce the occurrence of LI in elderly patients with hypertension [7]. Guo et al. (2021) showed that the changes of NLR, ANC, and WBC levels were independently and significantly correlated with the mRS score of patients with acute lacunar infarction, which can provide a reference for clinical evaluation of patients' prognosis [8]. The above research data study the prediction and analysis of the disease progression of different types of cerebral infarction from different research directions, but this study is to predict and analyze the disease progression of lacunar infarction from the active substances of endothelial cells in the focus. Ox-LDL is formed by a series of oxidative modifications of LDL. Under normal circumstances, LDL in plasma will not be oxidized, but if vascular endothelium is damaged, oxidation will be caused, and the oxidizing substances produced in the formation of Ox-LDL will damage endothelial cells, increase the permeability of endothelial cells, and make LDL easier to enter the subendothelial space. It causes the reduction of the synthesis of endothelial cell protective agent PGI2 and NO, which further aggravates the injury of endothelial cells, which is a vicious circle. NO is the most important vasodilator secreted by endothelial cells. PGI2 and NO have synergistic vasodilation, platelet aggregation prevention, and antithrombotic effects. The decrease of PGI2 and no will promote platelet aggregation and release oxygen ions [9–12].

The article "Predictive Analysis of Serum NO, PGI2, and Ox-LDL Levels on Disease Progression in Patients with Lacunar Cerebral Infarction" was retracted in 2023. Reasons: suspected computer-generated content; unreliable results or conclusions; concerns about the data; concerns about the results or conclusions.

The results of this study show that the levels of serum NO, PGI2, and Ox-LDL affect the progression of lacunar infarction. The levels of Ox-LDL in patients with lacunar infarction are at a high level, while the levels of serum NO and PGI2 are at a low level. The indexes of patients with progressive LI are significantly different from those of healthy people than those of patients with nonprogressive LI.

## 5. Summary

In this study, the factors affecting the progression of lacunar cerebral infarction were studied from the perspective of the changes of the levels of serum NO, PGI2, and Ox-LDL formed in endothelial cells. The above research data showed that compared with healthy people, patients with lacunar cerebral infarction had higher levels of Ox-LDL and lower levels of serum NO and PGI2, that is, the changes of serum NO, PGI2, and Ox-LDL levels in patients with lacunar cerebral infarction can be detected by endothelial function test, which can be widely used in clinical detection. However, there are still deficiencies in this study. Only the sample size of patients in our hospital is insufficient. In the follow-up, the number of samples will be increased for research, so as to obtain more accurate and credible conclusions.

## Figures and Tables

**Figure 1:** Comparison of general data of patients.

**Figure 2:** Comparison of serum NO, PGI2, and Ox-LDL levels between nonprogressive group and control group.

**Figure 3:** Comparison of serum NO, PGI2, and Ox-LDL levels between progression group and control group.

**Figure 4:** Comparison of serum NO, PGI2, and Ox-LDL levels between nonprogression group and progression group.

**Figure 5:** Comparison of serum NO, PGI2, and Ox-LDL levels in different groups.

**Table 1:** General clinical data of patients.

Classification of general clinical data		Number of people
Age	40-50	23 (16.67)
	50-60	47 (34.06)
	>60	68 (49.27)
Gender	Male	92 (66.67)
	Female	46 (33.33)
Degree of education	Primary school and below	32 (23.19)
	Junior high school	36 (26.09)
	High school and above	41 (29.71)
	Bachelor degree or above	29 (21.01)
Pathogenesis	Progressivity	67 (48.55)
	Nonprogressive	71(51.45)
*p* > 0.05		

**Table 2:** Scoring criteria of neurological deficit (NIHSS).

Item classification	Scoring criteria
Consciousness level	Awake = 0; lethargy = 1; drowsiness = 2; coma = 3
Awareness level questions (age, month)	Correct answers = 0; one item is correct = 1; incorrect or aphasia = 2
Consciousness level command (shaking hands, closing eyes)	All correct = 0; 1 correct = 1; all incorrect = 2
Gaze	Normal = 0; partial gaze paralysis = 1; complete gaze paralysis = 2
View	Normal = 0; partial hemianopia = 1; complete hemianopia = 2; bilateral hemianopia; double blind = 3
Facial paralysis	Normal = 0; paraplegia = 1; part = 2; complete = 3
Left (right) upper limb movement	Lift 90° or 45° for 10 s without falling = 0; the falling cannot be maintained for 10 s = 1; lifting cannot reach 90° or 45° = 2; unable to resist gravity and fall immediately = 3; no movement
Left (right) lower limb movement	Lift 30° and hold for 5S without falling = 0; falling nonimpact bed = 1; falling within 5S = 2; immediate drop = 3; no motion = 4
Limb ataxia	No ataxia = 0; one side = 1; on both sides = 2
Sensory deficit	None = 0; light to moderate = 1; completely missing = 2
Aphasia	None = 0; light to moderate = 1; severe aphasia = 2; complete aphasia or dumb = 3
Dysarthria	Normal = 0; light to moderate = 1; dumb or severe = 2
Ignore	Normal = 0; disappearance of bilateral stimulation = 1; severe partial neglect or more than one neglect = 2

The article "Predictive Analysis of Serum NO, PGI2, and Ox-LDL Levels on Disease Progression in Patients with Lacunar Cerebral Infarction" was retracted in 2023. Reasons: suspected computer-generated content; unreliable results or conclusions; concerns about the data; concerns about the results or conclusions.

**Table 3:** Comparison of serum NO, PGI2, and Ox-LDL between LI patients in nonprogression group and control group.

Group	*n*	Ox-LDL (U/L)	NO (ummol/L)	PGI2 (ng/L)
Nonprogress group	71	56.31 ± 2.6	75.74 ± 4.6	32.37 ± 2.8
Control group	34	45.67 ± 2.1	89.97 ± 3.1	36.48 ± 3.6
*t* value	—	1.012	0.817	3.567
*p* value	—	0.007	0.006	0.012

**Table 4:** Comparison of serum NO, PGI2, and Ox-LDL between LI patients in progression group and control group.

Group	*n*	Ox-LDL (U/L)	NO (ummol/L)	PGI2 (ng/L)
Progress group	67	79.46 ± 4.7	51.65 ± 5.2	27.21 ± 4.3
Control group	34	45.67 ± 2.1	88.97 ± 3.1	36.48 ± 3.6
*t* value	—	0.654	0.617	1.357
*p* value	—	0.003	0.004	0.011

**Table 5:** Comparison of serum NO, PGI2, and Ox-LDL between LI patients in progression group and nonprogression group.

Group	*n*	Ox-LDL (U/L)	NO (ummol/L)	PGI2 (ng/L)
Nonprogress group	71	56.31 ± 0	75.74 ± 4.6	32.37 ± 2.8
Progress group	67	79.46 ± 4.7	51.65 ± 5.2	27.21 ± 4.3
*t* value	—	1.267	1.038	1.204
*p* value	—	0.008	0.005	0.009

**Table 6:** Multivariate predictive analysis of disease progression in patients with lacunar infarction.

Observation index	Assignment	*β*	OR	95% CI	*p*
Ox-LDL	≤76.48 U/L	1.368	6.214	3.438-9.128	0.004
	>76.48 U/L				
NO	≤55.24 ummol/L	1287	3.671	1.957-5.497	0.009
	>55.24 ummol/L				
PGI2	≤29.78 ng/L	1.427	6.017	5.347-9.984	0.011
	>29.78 ng/L				

## Data Availability

The data underlying the results presented in the study are available within the manuscript.
